This article has been retracted.

# A Computational Model of Blood D-Dimer, Cystatin C, and CRP Levels Predicts the Risk of Intracranial Aneurysms and their Rupture

**DOI:** 10.1155/2022/2216509

**Published:** 2022-11-18

**Authors:** Liang Xing, Haibo Long, Rui Bo, Xue Gou, Yan He, Xing Peng

**Affiliations:** Department of Neurosurgery, Chongqing Hospital of Traditional Chinese Medicine, No. 6, Panxi Qizhi Road, Jiangbei District, Chongqing 400021, China

## Abstract

**Objective:**

The aim of this study is to construct a computational model of blood D-dimer, cystatin C, and CRP levels and to predict the risk of intracranial aneurysms and their rupture.

**Methods:**

A total of 69 intracranial aneurysms patients were selected as the case group, including 28 cases in the ruptured group and 41 cases in the unruptured group. Another 64 non-intracranial aneurysm patients were selected as the control group. The detection results of serum D-dimer, cystatin C, and CRP were collected. The logistic regression computational model was used to analyze the occurrence and risk factors of intracranial aneurysms. The receiver operating curves (ROC) of serum D-dimer, cystatin C, and C reactive protein (CRP) levels for predicting intracranial aneurysms and their rupture were drawn, and the area under the curve (AUC), sensitivity, and specificity were calculated.

**Results:**

The serum levels of D-dimer, cystatin C, and CRP in patients with intracranial aneurysms were significantly higher than those in the control group and the differences were statistically significant (*P* < 0.05). The serum levels of D-dimer, cystatin C, and CRP in patients with ruptured intracranial aneurysms were higher than those in patients with unruptured intracranial aneurysms, and the differences were also statistically significant (*P* < 0.05). The combined detection of serum D-dimer, cystatin C, and CRP levels has a higher AUC (0.9014) for predicting intracranial aneurysms and higher AUC (0.9412) for predicting ruptured intracranial aneurysms than D-dimer (0.7118 and 0.8750, respectively), cystatin C (0.6489 and 0.6180, respectively), and CRP (0.7764 and 0.6551, respectively) independent detection; the combined detection had a sensitivity of 93.75% and 87.80 for predicting the occurrence and rupture of intracranial aneurysms, and the specificity was 68.12% and 92.86%, respectively.

**Conclusion:**

The combined detection of serum D-dimer, cystatin C, and CRP levels is a very valuable indicator for predicting the occurrence and rupture of intracranial aneurysms, and combined detection can provide scientific evidence-based guidance for clinical prediction of the occurrence and rupture of intracranial aneurysms.

## 1. Introduction

Intracranial aneurysms is a disease mainly caused by congenital abnormality or acquired pathological damage of intracranial arteries [1]. The remodeling of the vascular wall leads to local expansion and deformation, resulting in the thinning of the vascular wall and the loss of the inner layer of elastic degradation. The probability of rupture and hemorrhage of the artery here will be much higher than that of normal intracranial vessels [2, 3]. Intracranial aneurysms are the main cause of approximately 85% of subarachnoid hemorrhages [4–6]. The 30-day mortality rate after aneurysmal subarachnoid hemorrhage can be as high as 45% [7]. Intracranial aneurysms have high morbidity, high disability, and high mortality and cause a serious burden on patients, their families, and society [8, 9]. Therefore, early prediction and prevention of the occurrence and rupture of intracranial aneurysms are of great value and significance.

D-dimer is a specific marker of the fibrinolytic process and its level is increased or positive is more common in secondary hyperfibrinolysis, such as hypercoagulable state, disseminated intravascular coagulation, kidney disease, organ transplant rejection reaction, and thrombolytic therapy. [10, 11]. Fukuda et al. [12] found that elevated D-dimer levels were significantly associated with intravascular embolization of aneurysms in patients with malformations complicated by subarachnoid hemorrhage. The value of serum D-dimer levels in the assessment of intracranial aneurysms occurrence and risk of rupture is currently unclear. Cystatin C is one of the cysteines cathepsin inhibitory proteins and is mainly used as a marker reflecting impaired renal function [13–15]. Cystatin C can potently inhibit cathepsin, and when the level of cystatin C decreases, the activity of cathepsin increases, which may lead to excessive decomposition of the extracellular matrix of the blood vessel wall, resulting in pathological damage [16–18]. According to research studies, there is also an imbalance between the cystatin C and cathepsin expression in isolated human intracranial aneurysms specimens [19, 20]. However, the value of cystatin C levels in the prediction and rupture risk assessment of intracranial aneurysms is currently unclear. C-reactive protein (CRP) is a functional protein that can immediately respond to the inflammatory state of the body. When the body is in an abnormal stress state such as infection, inflammatory response, and autoimmune disease, the inflammatory response to infection occurs and the body's autoimmune function is significantly reduced. The serum CRP level of the patient will increase rapidly due to the aggravation of the disease [21, 22]. Although related studies have reported the correlation of D-dimer, cystatin C, and CRP levels with intracranial aneurysms, it is still unclear whether these three indicators have the value of predicting the occurrence and rupture of intracranial aneurysms. Therefore, in this study, we planned to investigate the individual and combined indicators of D-dimer, cystatin C, and CRP levels in predicting the risk of intracranial aneurysms development and rupture.

## 2. Materials and Methods

### 2.1. Selection of Subjects

A total of 69 patients with intracranial aneurysms who were treated in Chongqing Hospital of Traditional Chinese Medicine from December 2018 to December 2021 were included in the case group. In addition, another 64 non-intracranial aneurysm patients were selected as the control group. Intracranial aneurysms were diagnosed by digital subtraction angiography, cranial CT angiography, or magnetic resonance angiography. Inclusion criteria were as follows: (1) Intracranial aneurysm and subarachnoid hemorrhage were diagnosed by 2 physicians through auxiliary examination. Exclusion criteria were as follows: (1) The diagnosis of intracranial aneurysms is unclear; (2) intracranial aneurysms combined with different cerebrovascular diseases, such as cerebral vascular occlusion, severe vascular stenosis, cerebral vascular malformation, and moyamoya disease; (3) associated with malignant tumor, metabolic disease, vascular inflammatory disease, systemic inflammation, etc.; (4) severe cardiovascular disease; (5) complicated with rheumatic immune diseases and hematopoietic system diseases; and (6) associated with other inflammatory diseases.

### 2.2. Methods

On the day of admission, about 5 ml of fasting venous blood was collected from the patients and the control group in the early morning, the plasma was separated after centrifuged at 4°C of 2000 r/min for 15 min. Plasma D-dimer and CRP levels were measured by chemiluminescence immunoassay, and cystatin C levels were measured by latex particle-enhanced immunoturbidimetry. All samples were tested in strict accordance with the kit instructions.

### 2.3. Statistical Analysis

The software used in this study was SPSS 26.0 (SPSS, Chicago, IL) and GraphPad prism (version 8.0, San Diego California, USA). Univariate analysis and multivariate analysis were performed to analyze the risk factors of intracranial aneurysms and their rupture, and the assignment results are shown in Table 1. The ROC of D-dimer, cystatin C, and CRP levels and combined detection indexes for the diagnosis of intracranial aneurysms and its rupture were drawn, and the AUC, sensitivity, specificity, and cutoff values were calculated. The significance level was *α* = 0.05, and *P* < 0.05 indicated that the difference was statistically significant.

## 3. Results

### 3.1. Comparison of Clinical Data between the Ruptured Group, The Unruptured Group, and the Control Group

The clinical data of the ruptured intracranial aneurysm group, the unruptured group, and the control group are shown in Table 2. A total of 69 patients with intracranial aneurysms, including 50 patients over the age of 60, only 19 patients under the age of 60, were selected. There were 22 males and 47 females, 38 patients with a history of hypertension, and 31 patients without a history of hypertension. There were 23 patients with a history of diabetes mellitus and 46 patients without a history of diabetes mellitus. Statistical analysis showed that there were statistically significant differences between the ruptured intracranial aneurysms group, the unruptured group, and the control group in age, the proportion of patients with a history of hypertension, and the proportion of patients with a history of diabetes mellitus (*P* < 0.05).

### 3.2. Correlation between the Serum D-Dimer Level and Intracranial Aneurysms and Their Rupture

The correlation between serum D-dimer levels and intracranial aneurysms were analyzed. The results showed that the level of serum D-dimer in patients with intracranial aneurysms was significantly higher than that in the control group, and the difference was extremely significant (*P* < 0.01, Figure 1(a)). In the patients with intracranial aneurysms, the serum D-dimer level in the ruptured group was significantly higher than that in the unruptured group, and the difference was statistically significant (*P* < 0.05, Figure 1(b)). We further used the receiver operating curve (ROC) to analyze the value of serum D-dimer in the diagnosis of intracranial aneurysms. The results showed that the AUC of serum D-dimer in the predicting intracranial aneurysms was 0.7118 (95% CI: 0.6214–0.8023, *P* < 0.001), the sensitivity was 95.31% (95% CI: 87.10%–98.72%), the specificity was 57.97% (95% CI: 46.21%–68.89%), and the cutoff value was 2.65 mg/L (Figure 1(c)). The AUC of serum D-dimer in predicting rupture risk of intracranial aneurysms was 0.8750 (95% CI: 0.7883–0.9617, *P* < 0.001), the sensitivity was 73.17% (95% CI: 58.07%–84.31%), the specificity was 96.43% (95% CI: 82.29%–99.82%), and the cutoff value was 4.02 mg/L (Figure 1(d)).

### 3.3. Correlation between the Serum Cystatin C Level and Intracranial Aneurysms and Rupture

We analyzed the correlation between serum cystatin C levels and intracranial aneurysms. The results showed that the level of serum cystatin C in patients with intracranial aneurysms was significantly higher than that in the control group and the difference was statistically significant (*P* < 0.05, Figure 2(a)). In the patients with intracranial aneurysms, the serum cystatin C level in the ruptured group was significantly higher than that in the unruptured group and the difference was statistically significant (*P* < 0.05, Figure 2(b)). We used receiver operating curve (ROC) analysis to analyze the value of serum cystatin C in predicting intracranial aneurysms. The results showed that the AUC of serum cystatin C for predicting intracranial aneurysms was 0.6489 (95% CI: 0.5448–0.7530, *P*=0.0031), the sensitivity was 53.13% (95% CI: 41.07%–64.82%), the specificity was 95.65% (95% CI: 87.98%–98.81%), and the cutoff value was 0.59 mg/L (Figure 2(c)). The AUC of serum cystatin C for predicting intracranial aneurysm rupture was 0.6180 (95% CI: 0.4830–0.7530, *P*=0.0978), the sensitivity was 97.56% (95% CI: 87.40%–99.87%), the specificity was 28.57% (95% CI: 15.25%–47.06%), and the cutoff value was 1.10 mg/L (Figure 2(d)).

### 3.4. Correlation between the Serum CRP Level and Intracranial Aneurysms and Rupture

We analyzed the correlation between serum CRP levels and intracranial aneurysms. The results showed that the level of serum CRP in patients with intracranial aneurysms was significantly higher than that in the control group, and the difference was statistically significant (*P* < 0.0001, Figure 3(a)). In the patients with intracranial aneurysms, the serum CRP level in ruptured patients was significantly higher than that in the unruptured group and the difference was statistically significant (*P* < 0.01, Figure 3(b)). We further used the ROC to analyze the value of serum CRP in the predicting intracranial aneurysms. The results showed that the AUC of serum CRP in the predicting intracranial aneurysms was 0.7764 (95% CI: 0.6913–0.8615, *P* < 0.001), the sensitivity was 93.75% (95% CI: 85.00%–97.54%), the specificity was 71.01% (95% CI: 59.43%–80.38%), and the cutoff value was 15.78 mg/L (Figure 3(c)). The AUC of serum CRP in predicting rupture of intracranial aneurysms was 0.6551 (95% CI: 0.5133–0.7968, *P* < 0.001), the sensitivity was 90.24% (95% CI: 77.45%–96.14%), the specificity was 42.86% (95% CI: 26.51%–60.93%), and the cutoff value was 60.74 mg/L (Figure 3(d)).

### 3.5. The Combined Detection Model of Serum D-Dimer, Cystatin C, and CRP Levels Predicted the Outcome of Intracranial Aneurysm and Rupture

Univariate analysis showed that age, history of hypertension, history of diabetes mellitus, high level of D-dimer, high level of cystatin C and high level of CRP in serum were risk factors for intracranial aneurysm (*P* < 0.05) (Table 3). The results of multivariate logistic regression analysis showed that high levels of D-dimer and high levels of cystatin C were independent risk factors for intracranial aneurysm (D-dimer: OR = 15.10, 95% CI: 3.08–74.02, *P* < 0.01; cystatin C: OR = 15.10, 95% CI: 3.08–74.02, *P* < 0.01) (Table 4). According to the results of logistic regression analysis, the AUC of the combined detection index for predicting the occurrence of intracranial aneurysms was 0.9014, the sensitivity was 93.75%, and the specificity was 68.12% (Figure 4(a)).

Univariate analysis showed that age, history of hypertension, history of diabetes mellitus, high level of D-dimer, high level of Cystatin C and high level of CRP in serum were risk factors for rupture of intracranial aneurysms (*P* < 0.05) (Table 5). The results of multivariate logistic regression analysis showed that high levels of D-dimer and high levels of cystatin C were independent risk factors for intracranial aneurysms (OR = 162.35, 95% CI: 12.26–2150.43, *P* < 0.01) (Table 6). According to the results of logistic regression analysis, the AUC of combined detection for predicting ROC in intracranial aneurysms was 0.9412, with a sensitivity of 87.80% and a specificity of 92.86% (Figure 4(b)).

The cutoff value of D-dimer was 4.02 mg/L, a low level indicated the D-dimer was less than 4.02 mg/L and a high level means D-dimer level was ≥4.02 mg/L. The cutoff value of cystatin C was 1.10 mg/L, a low level indicated the cystatin C < 1.10 mg/L, and high level means D-dimer level was ≥1.10 mg/L. The cutoff value of CRP was 60.74 mg/L, a low level indicated the CRP <60.74 mg/L and a high level means CRP level was ≥60.74 mg/L.

## 4. Discussion

Intracranial aneurysms are the main cause of subarachnoid hemorrhage, which can cause 30% to 50% of patients to die within the first 14 days after subarachnoid hemorrhage, and surviving patients will also have varying degrees of disability [4, 23, 24]. Studies have found that intracranial aneurysms can occur in people at any age and are more common in people aged 40 to 60, which has a serious impact on the lives of patients [25]. At present, an endovascular interventional therapy has been widely used in the treatment of intracranial aneurysms, which can effectively prevent intracranial aneurysms rupture and bleeding, and the postoperative mortality and morbidity rates of patients are low [26–28]. Although short-term data show promise for endovascular intervention, long-term follow-up data suggest that the incidence of incompletely embolized aneurysms requiring retreatment, residual aneurysm neck, and recurrent aneurysms cannot be ignored [27, 29, 30]. Rupture of an intracranial aneurysms can lead to a series of clinical symptoms, such as sudden explosive headache, nausea and vomiting, and disturbance of consciousness. At the same time, serious complications such as hydrocephalus, ischemic cerebral infarction, or vasospasm may occur, resulting in death of the patients [31, 32]. Therefore, looking for early diagnostic indicators and adopting clinical early intervention measures may be a new way to improve the poor clinical outcomes of patients with intracranial aneurysms [33].

D-dimer is a specific marker of fibrinolysis process, and its increased content or positive reflects the activation of the body's coagulation and fibrinolysis system [34]. D-dimer has been shown to be closely related to the prognosis of patients with coronary heart disease [35], sepsis [36], deep venous thrombosis [37], acute pulmonary embolism [38], and malignant cancer [39]. Fukuda et al. [11, 12] reported that elevated D-dimer levels in patients with acute subarachnoid hemorrhage were significantly associated with increased thromboembolic events during endovascular embolization of ruptured aneurysms. Hsu et al. [40] found that high plasma D-dimer levels could predict adverse outcomes in patients with acute ischemic stroke treated with intravenous thrombolysis. In this study, we found that serum D-dimer levels were elevated in patients with intracranial aneurysms, especially in ruptured patients. The reason may be due to the activation of coagulation and fibrinolysis systems in patients with ruptured intracranial aneurysms, and plasma D-dimer can just reflect the changes in coagulation and fibrinolysis, which will promote changes in blood system homeostasis, prone to thromboembolic events. Plasma D-dimer is a specific degradation product of cross-linked fibrin produced by the fibrinolytic system during coagulation and can be used as a molecular marker of hypercoagulability and hyperfibrinolysis in vivo. Increased plasma D-dimer levels reflect a hypercoagulable state and a high thrombus burden in patients, leading to an increased risk of thromboembolic events. Plasma D-dimer levels are closely related to focal vessel wall-associated fibrin formation, coagulation, and activity of unstable atherosclerotic plaques, and higher levels indicate an increased risk of thromboembolic events [11, 41].

Plasma cystatin C is a basic small molecule-secreted protein. As a cysteinase inhibitor, its main function is to regulate the activity of cysteinase, participate in the regulation of protein hydrolysis, and affect the degradation process of intracellular and extracellular matrix. Under the action of various injury factors such as hypertension and hyperlipidemia, vascular endothelial cells are first damaged, and then smooth muscle cells undergo changes such as proliferation and migration, and blood vessels begin to remodel. Eventually, atherosclerotic plaques or aneurysms form. This process involves the degradation and synthesis of cathepsin and there must be active expression of cathepsin, but the downregulation of Cystatin C, a cathepsin inhibitor, accelerates this process. Studies have shown that cystatin C is significantly related to the stability and regression of atherosclerotic plaques, the occurrence and development of heart disease and peripheral cardiovascular disease [42]. Abisi et al. [43] found that the expression level of cystatin C in the arterial wall of the aneurysm model was reduced. Lindholt et al. [44] further conducted a 3-year clinical observation on 151 patients with abdominal aortic aneurysm and found that serum cystatin C concentration was significantly negatively correlated with the size and annual expansion rate of abdominal aortic aneurysm. It is proved that the lack of cystatin C is closely related to the progression of aortic aneurysm, and we speculated that the lack of cystatin C cannot effectively inhibit the activity of cysteine protease. A study has found that in the late stage of aneurysm progression, the expression of cystatin C decreased with the progression of the aneurysm [45]. Our results also showed that cystatin C had a great potential in the prediction of intracranial aneurysms and its rupture. When predicting intracranial aneurysms alone, the specificity was as high as 95.65%, and the sensitivity was only 53.13%, the sensitivity of tumor rupture was as high as 97.56%, and the specificity was only 28.57%. This shows that cystatin C, as a protease inhibitor, participates in many pathological and physiological processes of the cardiovascular system and may become a molecular indicator for auxiliary diagnosis and detection in the occurrence and rupture of intracranial aneurysms.

C-reactive protein (CRP) is an acute-phase inflammatory factor closely related to the occurrence of cardiovascular and cerebrovascular diseases [46]. CRP is mainly synthesized in the liver and then released into the blood circulation after the induction of inflammatory factors. The serum CRP level in normal patients was very low. CRP is a functional protein that can immediately respond to the inflammatory state of the body. When the body is in an abnormal stress state such as infection, inflammatory response, and autoimmune disease, the inflammatory response to infection occurs, the body's autoimmune function is significantly reduced, and the serum CRP level of the patient will increase rapidly due to the aggravation of the disease [47]. CRP has been used as a biomarker for diagnosing and monitoring infections and proliferative diseases in patients and has an important role in assessing the severity of the disease [48].

No study has reported the correlation between the occurrence and rupture of intracranial aneurysms and the above indicators. Therefore, this study we analyzed the value of serum D-dimer, cystatin C, and CRP in the diagnosis of the occurrence and rupture of intracranial aneurysms alone and in combination. In this study, we found that the combined detection of D-dimer, cystatin C, and CRP had a sensitivity of 93.75% and a specificity of 68.12% for the diagnosis of intracranial aneurysms; the sensitivity was as high as 87.80%, and the specificity was as high as 92.86%. It is suggested that the combination of D-dimer, cystatin C, and CRP detection has a high application value as an auxiliary diagnostic tool for the occurrence and rupture of intracranial aneurysms.

This study also has some limitations. First, the sample size included in this study is relatively small, and further verification is required in a larger sample. Second, if the correlation between these indicators and the prognosis of patients with intracranial aneurysms can be further studied, it will further enhance the value of this study. In addition, the correlation of these indicators with the pathogenesis of intracranial aneurysms needs to be further studied in in vitro and in vivo models.

## 5. Conclusion

The results of our study prove that the combined detection of serum D-dimer, cystatin C, and CRP levels is a very valuable indicator for predicting the occurrence and rupture of intracranial aneurysms and can be used for clinical diagnosis of the occurrence and rupture of intracranial aneurysms. This study can provide scientific evidence-based guidance for clinical diagnosis of the occurrence and rupture of intracranial aneurysms.

## Figures and Tables

**Figure 1:** Correlation of serum D-dimer levels with intracranial aneurysms and rupture. (a) Comparison of serum D-dimer levels between patients with intracranial aneurysms and controls. (b) Comparison of serum D-dimer levels in intracranial aneurysms patients with ruptured and unruptured groups. (c) Receiver operating curve (ROC) of serum D-dimer levels for the diagnosis of intracranial aneurysms. (d) Receiver operating curve (ROC) of serum D-dimer levels predicting rupture of intracranial aneurysms. Statistical analysis was performed using *t*-test, ^*∗*^*P* < 0.05, ^*∗∗∗∗*^*P* < 0.0001.

**Figure 2:** Correlation of serum cystatin C levels with intracranial aneurysms and rupture. (a) Comparison of serum cystatin C levels between patients with intracranial aneurysms and controls. (b) Comparison of serum cystatin C levels in intracranial aneurysms patients with ruptured and unruptured. (c) Receiver operating curve (ROC) of serum cystatin C levels for predicting intracranial aneurysms. (d) Receiver operating curve (ROC) of serum cystatin C levels predicting rupture of intracranial aneurysms. Statistical analysis was performed using *t*-test, ^*∗*^*P* < 0.05.

**Figure 3:** Correlation of serum C reactive protein (CRP) levels with intracranial aneurysms and rupture. (a) Comparison of serum CRP levels between patients with intracranial aneurysms and controls. (b) Comparison of serum CRP levels in intracranial aneurysms patients with ruptured and unruptured groups. (c) Receiver operating curve (ROC) of serum CRP levels for the predicting intracranial aneurysms. (d) Receiver operating curve (ROC) of serum CRP levels predicting rupture of intracranial aneurysm. Statistical analysis was performed using *t*-test,  ^*∗*^ ^*∗*^*P* < 0.01,  ^*∗*^ ^*∗*^ ^*∗*^ ^*∗*^*P* < 0.0001.

**Figure 4:** Correlation of combined detection of serum D-dimer, cystatin C, and C reactive protein (CRP) levels with intracranial aneurysms and rupture. (a) Receiver operating curve (ROC) of combined detection of serum D-dimer, cystatin C, and CRP levels in predicting intracranial aneurysm. (b) Receiver operating curve (ROC) of combined detection of serum D-dimer, cystatin C, and CRP levels in predicting rupture of intracranial aneurysms.

**Table 1:** Logistic regression analysis assignments.

Index	Assignment result
*Age (years)*	
<60	1
≥60	2

*Sex*	
Male	1
Female	2

*History of hypertension*	
Yes	1
No	2

*History of diabetes mellitus*	
Yes	1
No	2

**Table 2:** Comparison of clinical data of the ruptured intracranial aneurysm group, unruptured group, and control group.

	Intracranial aneurysm			Control group (*n* = 64)	*P* value
	Total (*n* = 69)	Ruptured group (*n* = 28)	Unruptured group (*n* = 41)		
*Age (years, n(%))*					
<60	19 (27.54%)	3 (10.71%)	16 (39.02%)	33 (51.56%)	0.001
≥60	50 (72.46%)	25 (89.29%)	25 (60.98%)	31 (48.44%)	

*Sex(n(%))*					
Male	22 (31.88%)	7 (25.00%)	15 (36.59%)	22 (34.38%)	0.576
Female	47 (68.12%)	21 (75.00%)	26 (63.41%)	42 (65.63%)	

*History of hypertension (n(%))*					
Yes	38 (55.07%)	22 (78.57%)	16 (39.02%)	7 (10.94%)	<0.001
No	31 (44.93%)	6 (21.43%)	25 (60.98%)	57 (89.06%)	

*History of diabetes mellitus (n(%))*					
Yes	23 (33.33%)	14 (50.00%)	9 (21.95%)	10 (15.63%)	0.002
No	46 (66.67%)	14 (50.00%)	32 (78.05%)	54 (84.38%)	

**Table 3:** Univariate analysis of intracranial aneurysms.

	Intracranial aneurysm (*n* = 69)	Control group (*n* = 64)	*χ * ^2^ value	*P* value
*Age (years, n(%))*				
<60	19 (27.54%)	33 (51.56%)	8.049	0.005
≥60	50 (72.46%)	31 (48.44%)		

*Sex (n(%))*				
Male	22 (31.88%)	22 (34.38%)	0.093	0.760
Female	47 (68.12%)	42 (65.63%)		

*History of hypertension (n(%))*				
Yes	38 (55.07%)	7 (10.94%)	28.890	<0.001
No	31 (44.93%)	57 (89.06%)		

*History of diabetes mellitus (n(%))*				
Yes	23 (33.33%)	10 (15.63%)	5.581	0.018
No	46 (66.67%)	54 (84.38%)		

*D-dimer*				
Low level	29 (42.03%)	61 (95.31%)	43.088	<0.001
High level	40 (57.97%)	3 (4.69%)		

*Cystatin C*				
Low level	3 (4.35%)	34 (53.13%)	39.341	<0.001
High level	66 (95.65%)	30 (46.88%)		

*CRP*				
Low level	30 (43.48%)	60 (93.75%)	38.355	<0.001
High level	39 (56.52%)	4 (6.25%)		

**Table 4:** Multivariate logistic regression analysis of intracranial aneurysms.

	B	S.E	Wald	df	Sig	Exp (B)	95% C.I. for EXP (B)
Age ≥60	0.13	0.55	0.06	1.00	0.81	1.14	0.39–3.39
Sex	−0.12	0.55	0.05	1.00	0.83	0.89	0.31–2.59
History of hypertension	−1.25	0.71	3.12	1.00	0.08	0.29	0.07–1.15
History of diabetes mellitus	−0.90	0.85	1.12	1.00	0.29	0.41	0.08–2.15
D-dimer high level	2.72	0.81	11.20	1.00	<0.01	15.10	3.08–74.02
Cystatin C high level	3.20	0.80	16.10	1.00	<0.01	24.52	5.14–116.97
CRP high level	0.99	1.14	0.76	1.00	0.38	2.70	0.29–25.02
Constant	−3.29	1.28	6.61	1.00	0.01	0.04	

**Table 5:** Univariate analysis of intracranial aneurysm rupture.

	Rupture group (*n* = 28)	Unruptured group (*n* = 41)	Χ^2^ value	*P* value
*Age (years, n(%))*				
<60	3 (10.71%)	16 (39.02%)	6.683	0.010
≥60	25 (89.29%)	25 (60.98%)		

*Sex(n(%))*				
Male	7 (25.00%)	15 (36.59%)	1.028	0.311
Female	21 (75.00%)	26 (63.41%)		

*History of hypertension (n(%))*				
Yes	22 (78.57%)	16 (39.02%)	10.517	0.001
No	6 (21.43%)	25 (60.98%)		

*History of diabetes mellitus (n(%))*				
Yes	14 (50.00%)	9 (21.95%)	5.890	0.015
No	14 (50.00%)	32 (78.05%)		

*D-dimer*				
Low level	1 (3.57%)	30 (73.17%)	32.573	<0.001
High level	27 (96.43%)	11 (26.83%)		

*Cystatin C*				
Low level	20 (71.43%)	40 (97.56%)	10.017	0.002
High level	8 (28.57%)	1 (2.44%)		

*CRP*				
Low level	16 (57.14%)	37 (90.24%)	10.235	0.001
High level	12 (42.86%)	4 (9.76%)		

**Table 6:** Multivariate logistic regression analysis of intracranial aneurysms rupture.

	B	S.E.	Wald	df	Sig.	Exp (B)	95% C.I. for EXP (B)
Age ≥60	2.11	1.26	2.79	1.00	0.10	8.23	0.70–97.38
Male	0.67	1.09	0.38	1.00	0.54	1.95	0.23–16.46
History of hypertension	−0.16	1.15	0.02	1.00	0.89	0.86	0.09–8.08
History of diabetes mellitus	−0.56	1.16	0.24	1.00	0.63	0.57	0.06–5.49
D-dimer high level	5.09	1.32	14.91	1.00	<0.01	162.35	12.26–2150.43
CRP high level	2.06	1.25	2.71	1.00	0.10	7.82	0.68–90.39
Constant	−27.17	21240.47	<0.01	1.00	1.00	<0.01	

The analysis of cystatin C showed *P*=1.0, which is not shown in the table here.

## Data Availability

The data used to support the findings of this study are available from the corresponding author upon request.
